The article "Effects of Ulinastatin on Myocardial Ischemia-Reperfusion Injury, Cardiac Function, and Serum TNF-α and IL-10 Levels in Patients Undergoing Cardiac Valve Replacement under Cardiopulmonary Bypass" was retracted in 2023. Reasons: signs of a paper mill; suspected computer-generated content; unreliable results or conclusions; concerns about the data.

# Effects of Ulinastatin on Myocardial Ischemia-Reperfusion Injury, Cardiac Function, and Serum TNF-*α* and IL-10 Levels in Patients Undergoing Cardiac Valve Replacement under Cardiopulmonary Bypass

**DOI:** 10.1155/2022/1823398

**Published:** 2022-04-01

**Authors:** Hai Wang, Dafa Zhang, Hongbo Qian, Jun Nie, Jun Wei

**Affiliations:** Department of Cardiovascular Surgery, Yijishan Hospital, The First Affiliated Hospital of Wannan Medical College, Wuhu City, 241000 Anhui Province, China

## Abstract

**Background:**

Myocardial ischemia-reperfusion injury (MIRI) is a very common adverse reaction after cardiac valve replacement (CVR) under cardiopulmonary bypass, which seriously affects the rehabilitation and prognosis of patients.

**Objective:**

The prevention and treatment of MIRI are a hotspot of modern medical research, and this study is aimed at providing reliable reference and guidance for future clinical prevention and treatment of MIRI by analyzing the effects of ulinastatin (UL) on cardiac function and MIRI of patients after CVR.

**Methods:**

A total of 104 patients undergoing CVR under cardiopulmonary bypass in our hospital were selected as research participants. Among them, 52 patients treated with UL were assigned to the observation group, and the rest 52 patients given the same amount of normal saline were assigned to the control group. The cardiopulmonary bypass status, postoperative status, cardiac function, inflammatory response, oxidative stress response, and hemodynamics were observed and compared between the two groups. In addition, clinical efficacy and safety and patient prognosis were compared.

**Results:**

Through experimental analysis, we found that UL had no significant effect on the clinical efficacy, safety, and prognosis of patients after surgery (*P* > 0.05) but had obvious protective effects on cardiopulmonary bypass status, cardiac function, inflammation, oxidative stress, and hemodynamics (*P* < 0.05).

**Conclusion:**

UL can effectively prevent the occurrence of MIRI after CVR under cardiopulmonary bypass, which is worthy of clinical application.

## 1. Introduction

Clinically, myocardial ischemia-reperfusion injury (MIRI) is a very common cardiovascular disease, mainly due to the fact that although the ischemic myocardium restores its normal perfusion capacity after acute coronary occlusion and recanalization, its tissue damage is progressively aggravated [1]. MIRI is a common complication after open heart surgery, with an incidence rate as high as 8%-15% [2]. At present, its pathogenesis has not been fully clarified, but calcium overload, energy metabolism disorder, increased oxygen free radicals, and intensified inflammatory response are considered to be the key factors of MIRI [3, 4]. MIRI is mainly manifested as intermittent pain, which may be accompanied by shock and heart failure in severe cases, and even sudden cardiac death without timely treatment, endangering the life of patients [5, 6]. According to one study [7], over 20% of patients die due to MIRI during surgery; so, its potential threat must be taken seriously by patients and clinical staff. This study mainly analyzes the types of surgeries that can prevent surgery-related MIRI, which has important implications for improving patient outcomes and reducing patient mortality.

The article "Effects of Ulinastatin on Myocardial Ischemia-Reperfusion Injury, Cardiac Function, and Serum TNF-α and IL-10 Levels in Patients Undergoing Cardiac Valve Replacement under Cardiopulmonary Bypass" was retracted in 2023. Reasons: signs of a paper mill; suspected computer-generated content; unreliable results or conclusions; concerns about the data.

Cardiac valve replacement (CVR) under cardiopulmonary bypass is the most common type of cardiovascular surgery. It can restore the impaired blood perfusion ability of patients through artificial heart valves, contributing to good hemodynamic characteristics and a very low incidence of thrombosis [8, 9]. At the current stage, CVR under cardiopulmonary bypass is widely used in clinical practice, which is effective in the treatment of rheumatic valvular disease, valvular heart disease, and others. However, it is likely to give rise to MIRI because of occlusion and reopening of aorta during the procedure, which may lead to serious postoperative adverse reactions [10–12]. Currently, searching solutions to MIRI after CVR under cardiopulmonary bypass have become a major clinical research hotspot [13], but no remarkable achievements have been hotspot so far. Ulinastatin (UL), a protease inhibitor, is a glycoprotein extracted from fresh urine that can inhibit the activity of a variety of proteolytic enzymes. Originally used for the treatment of recurrent pancreatitis, it has been later confirmed to have excellent rescue effects in acute circulatory failure [14]. Recently, UL has been shown to be effective in improving the hemodynamics and reducing the occurrence of reperfusion injury in patients undergoing percutaneous coronary intervention [15]. Based on this, Liu et al. and Zhao et al. found that UL showed a stable protective effect in animal models of spinal cord MIRI and liver MIRI [16, 17]. However, the effect of UL on MIRI after CVR under cardiopulmonary bypass has not been clarified and needs further confirmation.

In view of the increasing potential risks of MIRI, this study analyzed the effects of UL on cardiac function and MIRI of patients after CVR under cardiopulmonary bypass, so as to provide reliable reference and guidance for future clinical prevention and treatment of MIRI.

## 2. Materials and Methods

### 2.1. Patient Information

A total of 104 patients who underwent CVR under cardiopulmonary bypass in Yijishan Hospital, the First Affiliated Hospital of Wannan Medical College from March 2020 to February 2021 were enrolled for prospective analysis. According to the difference in intervention methods, 52 cases treated with UL were included in the observation group (Obs group), while the other 52 cases treated with the same amount of normal saline were included in the control group (Con group). This experiment was approved by the ethics committee of our hospital, and all the enrolled participants signed the informed consent.

The article "Effects of Ulinastatin on Myocardial Ischemia-Reperfusion Injury, Cardiac Function, and Serum TNF-α and IL-10 Levels in Patients Undergoing Cardiac Valve Replacement under Cardiopulmonary Bypass" was retracted in 2023. Reasons: signs of a paper mill; suspected computer-generated content; unreliable results or conclusions; concerns about the data.

### 2.2. Inclusion and Exclusion Criteria

Inclusion criteria were as follows: patients diagnosed with congenital heart valve disease, degenerative disease, or rheumatic valvular disease; patients who meet the indications for CVR; patients who underwent cardiac mitral valve replacement or cardiac tricuspid valve replacement under valve cardiopulmonary bypass; patients > 18 years old; and patients with New York Heart Association (NYHA) functional classification grade III-IV. Exclusion criteria were as follows: patients with drug allergy, patients with a history of other cardiac surgery, patients with multiple cardiovascular or cerebrovascular diseases, and patients with organ or immune dysfunction.

### 2.3. Surgery Method

CVR under cardiopulmonary bypass of all the enrolled patients was completed by the same surgical team of our hospital. Specifically, before surgery, each patient was given basic treatment such as diuresis and cardiac strengthen measures. After routine thoracotomy, 3 mg/kg heparin (Qilu Pharmaceutical Co., Ltd., State Food and Drug Administration (SFDA) Approval No.: H20030428) was injected intravenously. Cardiopulmonary bypass was established after 480 s of activated coagulation: Intubations were placed in the superior and inferior vena cava and aorta, and a catheter was inserted into the left atrium. The temperature was controlled at (30 ± 2)°C, and the superior and inferior vena cava was separated from the aorta. The aortic root was intermittently perfused with 4°C cardioplegia at an initial dose of 20 mL/kg, followed by 10 m/kg at 20-30 min intervals. The diseased valve tissue was excised through the interatrial septum, and the prosthetic valve was closed with mattress suture. Electrocardiogram (ECG) monitoring was performed after surgery to pay close attention to patients' vital signs and maintain circulatory system stability. In addition, pH values were monitored regularly, and antibiotics, polarized liquid, and other related treatments were given. Among them, in the cardioplegia injected into patients, 10,000 U/kg UL was added for the observation group, while the same amount of normal saline was added for the control group.

The article "Effects of Ulinastatin on Myocardial Ischemia-Reperfusion Injury, Cardiac Function, and Serum TNF-α and IL-10 Levels in Patients Undergoing Cardiac Valve Replacement under Cardiopulmonary Bypass" was retracted in 2023. Reasons: signs of a paper mill; suspected computer-generated content; unreliable results or conclusions; concerns about the data.

### 2.4. Sample Collection

Venous blood was sampled from each patient before surgery (T0), at 8 h after surgery (T1) and at 24 h after surgery (T2). Then, the levels of creatine kinase MB (CK-MB) and cardiac troponin I (cTnI) in the samples were determined via an automatic biochemistry analyzer with kits purchased from Immunotech Co., Ltd. and Beckman Coulter (USA) Co., Ltd., respectively. In addition, the levels of tumor necrosis factor-*α* (TNF-*α*), interleukin-10 (IL-10), superoxide dismutase (SOD), and malondialdehyde (MDA) were detected via enzyme-linked immunosorbent assay (ELISA) with kits all purchased from Chongqing Zhongyuan Huiji Biotechnology Co., Ltd. Moreover, stroke volume index (SVI), pulmonary arterial wedge pressure (PAWP), and left ventricular stroke work index (LVSWI) of each patient were determined via a hemodynamic monitor (LIDCO, UK, HM 81-01).

### 2.5. Follow-Up for Prognosis

Patients in both groups were followed up for 6 months through hospital reexamination, to record disease recurrence and evaluate their quality of life using the Medical Outcomes Study (MOS) 36-Item Short-Form Health Survey (SF-36). The MOS SF-36 is scored on a scale of 0-100, with higher scores indicating better quality of life.

### 2.6. Efficacy Assessment

Markedly effective was as follows: the NYHA classification was grade I or was improved by 2 grades or more. Effective was as follows: the NYHA classification was improved by 1 grade. Ineffective was as follows: The NYHA classification was not improved or increased from grade IV to grade III: total effective rate = (the number of cases with markedly effective treatment + the number of cases with effective treatment)/total number of cases × 100%.

### 2.7. Outcome Measures

Cardiopulmonary bypass status was as follows: aortic crossclamp time, cardiopulmonary bypass time, and auxiliary cardiopulmonary bypass time; postoperative status was as follows: cardiac autorebeating rate, pacemaker utilization rate, electrical defibrillation rate, dopamine utilization rate, and adrenaline utilization rate; cardiac function was as follows: CK-MB and cTnI levels; inflammatory reaction was as follows: TNF-*α* and IL-10 levels; oxidative stress reaction was as follows: MDA and SOD levels; hemodynamics was as follows: PAWP, LVSWI, and SVI; clinical efficacy and safety; prognosis was as follows: disease recurrence rate and SF-36 score.

### 2.8. Statistical Analyses

This study adopted SPSS22.0 for statistical analyses. Enumeration data such as sex were expressed as (*n*/%) and analyzed via the chi-square test. Measurement data such as cTnl were expressed as (^−^*χ* ± *s*). Independent samples *t*-test was used for data comparison between the two groups, paired *t*-test was used for intragroup comparisons before and after treatment, and one-way analysis of variance (ANOVA) as well as LSD post hoc test was used for multigroup comparisons. *P* < 0.05 indicates a remarkable difference.

The article "Effects of Ulinastatin on Myocardial Ischemia-Reperfusion Injury, Cardiac Function, and Serum TNF-α and IL-10 Levels in Patients Undergoing Cardiac Valve Replacement under Cardiopulmonary Bypass" was retracted in 2023. Reasons: signs of a paper mill; suspected computer-generated content; unreliable results or conclusions; concerns about the data.

## 3. Results and Discussion

### 3.1. Clinical Baseline Data of the Two Groups Were Not Significantly Different

The two groups showed no significant difference in clinical baseline data (*P* > 0.05, Table 1).

### 3.2. The Obs Group Has Superior Cardiopulmonary Bypass Status to the Con Group

The Obs group experienced shorter aortic crossclamp time, cardiopulmonary bypass time, and auxiliary cardiopulmonary bypass time than the Con group (all *P* < 0.05, Figure 1).

### 3.3. The Obs Group Showed Better Postoperative Status than the Con Group

After surgery, the two groups presented no significant difference in cardiac autorebeating rate and pacemaker utilization rate (both *P* > 0.05), but the Obs group showed lower electrical defibrillation rate, dopamine utilization rate, and adrenaline utilization rate than the Con group (all *P* < 0.05) (Table 2).

### 3.4. The Obs Group Showed Better Cardiac Function than the Con Group

At T0, the levels of CK-MB and cTnI were not significantly different between the two groups (both *P* > 0.05); but at T1 and T2, the Obs group showed lower levels of CK-MB and cTnI than the Con group (both *P* < 0.05). In both groups, the levels of CK-MB and cTnI increased at T1, but decreased at T2 (both *P* < 0.05) (Figure 2).

### 3.5. The Obs Group Showed Milder Inflammation than the Con Group

There were no significant differences in TNF-*α* and IL-10 levels between the two groups at T0 (both *P* > 0.05); at T1 and T2, the Obs group showed a lower TNF-*α* level and a higher IL-10 level than the Con group (both *P* < 0.05). In addition, the TNF-*α* level of both groups increased at T1 but decreased at T2, while the IL-10 level decreased at T1 and increased at T2 (both *P* < 0.05) (Figure 3).

### 3.6. The Obs Group Showed Milder Oxidative Stress Reaction than the Con Group

At T0, no significant difference was found between the two groups in MDA and SOD (both *P* > 0.05); at T1 and T2, the Obs group showed a lower MDA level and a higher SOD level than the Con group (both *P* < 0.05). In both groups, the MDA level increased at T1 but decreased at T2, while the SOD level decreased at T1 and increased at T2 (both *P* < 0.05) (Figure 4).

### 3.7. Hemodynamics of the Obs Group Was Superior to That of the Con Group

The two groups were not significantly different in PAWP and SVI at T0, T1, and T2, as well as LVSWI at T0 (all *P* > 0.05); at T1 and T2, the Obs group showed a higher LVSWI level than the Con group (both *P* < 0.05). In both groups, PAWP decreased with time and LVSWI increased with time, while SVI decreased at T1 and increased at T2 (all *P* < 0.05) (Figure 5).

The article "Effects of Ulinastatin on Myocardial Ischemia-Reperfusion Injury, Cardiac Function, and Serum TNF-α and IL-10 Levels in Patients Undergoing Cardiac Valve Replacement under Cardiopulmonary Bypass" was retracted in 2023. Reasons: signs of a paper mill; suspected computer-generated content; unreliable results or conclusions; concerns about the data.

### 3.8. Clinical Efficacy and Safety Were Not Significantly Different between the Two Groups

No significant difference was detected between Obs group and Con group in total effective rate (90.38% vs. 86.54%, *P* > 0.05) nor in the incidence of adverse reactions (7.68% vs. 11.54%, *P* > 0.05) (Table 3).

### 3.9. Patient Prognosis Rate Was Not Significantly Different between the Two Groups

During the 6 months follow-up for prognosis judgment, 48 patients in the Obs group and 49 patients in the Con group were successfully followed up. There was no significant difference in one-year disease recurrence rate and quality of life score between the two groups (both *P* > 0.05) (Figure 6).

## 4. Discussion

MIRI is a great potential threat, as it seriously affects the patient's heart function and postoperative rehabilitation and worsens their prognosis [18, 19]. Searching for measures to prevent MIRI after CVR is a clinical research hotspot at present. For instance, LV et al. proposed that the application of UL can effectively prevent the occurrence of cerebral ischemia-reperfusion injury [20]. However, due to the lack of relevant clinical studies, the application effect of UL in CVR is still controversial. In this study, the application value of UL is investigated from multiple perspectives, aimed at providing more accurate guidance and suggestions for the prevention and treatment of MIRI during CVR under cardiopulmonary bypass in the future.

Some researchers have analyzed the protective effect or mechanism of UL in MIRI. For example, Kawamura et al. [21] reported that UL plays a cardioprotective role in MIRI related to open heart surgery with cardiopulmonary bypass by inhibiting the release of IL-8 and IL-6. Yang et al. [22] proposed that UL can protect cardiac function by downregulating the expression of TNF-*α* and inhibiting MIRI induced by c-Jun N-terminal kinase (JNK) and P38 mitogen-activated protein kinase (MAPK) signaling pathways. The results of this study showed that the application of UL in has no significant effect on the clinical efficacy, safety, and prognosis of patients undergoing CVR under cardiopulmonary bypass, but it had significant protective effects on patients' cardiopulmonary bypass status, cardiac function, inflammation, oxidative stress, and hemodynamics. Evidence has shown that during the development of MIRI, the infiltration ability of neutrophils will be greatly enhanced, which mediates the aggravation of inflammatory injury of myocardial tissue and generates massive oxygen free radicals to induce the peroxidation of a large number of cells and the consequent denaturation of enzymes and ion channel proteins and DNA chain breakage, resulting in injury of myocardial tissue and myocardial function [23]. In addition, MIRI can also inhibit adenosine triphosphate (ATP), which reduces the transduction ability of calcium ions, resulting in calcium overload and calcification damage in cells [24]. Therefore, the key to the prevention and treatment of MIRI lies in the elimination of oxygen free radicals on the one hand and the acceleration of calcium ion transduction on the other. When Fei et al. conducted pharmacological analysis of UL, they found that both ends of UL had negatively charged polar molecules, which could closely bind to phospholipid molecules on the surface of myocardial cell membrane to maintain the stability of cell membrane, thus improving the body's cardiopulmonary bypass [25]. In addition, UL can provide energy for myocardial cells and relieve the enzymatic hydrolysis of myocardium, thereby reducing the release of oxygen free radicals and alleviating intracellular calcium overload to improve cardiac function, which can be fully confirmed by the results of this experiment and previous studies [26, 27]. UL can act as a calcium antagonist of cells and block the activation of calmodulin, the calcium ion protein, to reduce the occurrence of inflammatory injury and immune injury [28]. In addition, as a protease inhibitor, UL is a very classic oxygen free radical scavenger. When UL is hydrolyzed, it can release energy exceeding ATP, transfer phosphate groups to cell molecules, and restore the original ability of cells [22, 29]. Moreover, UL can increase the phosphoric acid activity of cells while reducing endothelial cell tension, so as to improve microcirculation and hemodynamics [30].

The article "Effects of Ulinastatin on Myocardial Ischemia-Reperfusion Injury, Cardiac Function, and Serum TNF-α and IL-10 Levels in Patients Undergoing Cardiac Valve Replacement under Cardiopulmonary Bypass" was retracted in 2023. Reasons: signs of a paper mill; suspected computer-generated content; unreliable results or conclusions; concerns about the data.

Through previous studies, we found that the combination of different anesthetic and sedative drugs with UL can improve the ability of UL for the management and treatment of MIRI [31, 32], which would be one of the focuses of our follow-up research. In addition, expanded sample size is needed to analyze the prevention and treatment of MIRI after other open heart surgeries with UL. Moreover, a longer prognostic follow-up of patients enrolled in this study is needed to obtain more comprehensive experimental results for clinical reference.

## 5. Conclusion

UL can effectively prevent and treat MIRI after CVR under cardiopulmonary bypass and improves the cardiopulmonary bypass status, cardiac function, inflammatory response, oxidative stress response, and hemodynamics of patients, which is worthy of clinical application.

## Figures and Tables

**Figure 1:** Comparison of cardiopulmonary bypass status. (a) Cardiopulmonary bypass time. (b) Aortic crossclamp time. (c) Auxiliary cardiopulmonary bypass time. #*P* < 0.05.

**Figure 2:** Comparison of cardiac function. (a) CK-MB level. (b) cTnI level vs. T0, #*P* < 0.05 vs. T1, &*P* < 0.05 vs. Obs group, ^∗^*P* < 0.05.

**Figure 3:** Comparison of Inflammatory reaction. (a) TNF-*α* level. (b) Il-10 level vs. T0, #*P* < 0.05 vs. T1, &*P* < 0.05 vs. Obs group, ^∗^*P* < 0.05.

**Figure 4:** Comparison of oxidative stress reaction. (a) MDA level. (b) SOD level vs. T0, #*P* < 0.05 vs. T1, &*P* < 0.05 vs. Obs group, ^∗^*P* < 0.05.

**Figure 5:** Comparison of emodynamics. (a) PAWP level. (b) LVSWI level. (c) SVI level vs. T0, #*P* < 0.05 vs. T1, &*P* < 0.05 vs. Obs group, ^∗^*P* < 0.05.

**Figure 6:** Comparison of prognosis. (a) Disease recurrence rate. (b) SF-36 score.

**Table 1:** Clinical baseline data (*n* (%)).

	Obs group	Con group	*t*/*χ*^2^	*P*
Age	54.6 ± 8.7	53.5 ± 7.4	0.695	0.489
Gender			0.369	0.543
Male	31 (59.62)	34 (65.38)		
Female	21 (40.38)	18 (34.62)		
Type of disease			0.378	0.828
Congenital heart valve disease	17 (32.69)	20 (38.46)		
Degenerative disease	13 (25.00)	12 (23.08)		
Rheumatic valvular disease	22 (42.31)	20 (38.46)		
Type of surgery			0.175	0.676
Tricuspid valve replacement	18 (34.62)	16 (30.77)		
Mitral valve replacement	34 (65.38)	36 (69.23)		
Valve type			0.633	0.426
Mechanical valve	42 (80.77)	45 (86.54)		
Biological valve	10 (19.23)	7 (13.46)		
Family history of illness			0.377	0.539
Have	7 (13.46)	5 (9.62)		
None	45 (86.54)	47 (90.38)		
Smoking			0.650	0.420
Yes	22 (42.31)	18 (34.62)		
No	30 (57.69)	34 (65.38)		
Drinking			0.046	0.830
Yes	16 (30.77)	15 (28.85)		
No	36 (69.23)	37 (71.15)		
Living environment			0.633	0.426
City	42 (80.77)	45 (86.54)		
Countryside	10 (19.23)	7 (13.46)		

**Table 2:** Comparison of postoperative status (*n* (%)).

	Autoresuscitation	Electric defibrillation	Use pacemaker	Use dopamine	Use adrenaline
Obs group	52 (100.0)	5 (9.62)	1 (1.92)	24 (46.15)	3 (5.77)
Con group	52 (100.0)	15 (28.85)	2 (3.85)	36 (69.23)	10 (19.23)
*χ* ^2^	—	6.190	0.343	5.673	4.308
*P*	—	0.013	0.558	0.017	0.038

**Table 3:** Comparison of clinical efficacy and safety (*n* (%)).

	Obs group	Con group	*χ* ^2^	*P*
Total effective rate (%)	90.38	86.54	0.377	0.539
Significant	30 (57.69)	26 (50.00)		
Efficient	17 (32.69)	19 (36.54)		
Invalid	5 (9.62)	7 (13.46)		
Total incidence (%)	7.68	11.54	0.443	0.506
Lung infection	1 (1.92)	1 (1.92)		
Atelectasis	1 (1.92)	2 (3.85)		
Impairment of shoulder mobility	1 (1.92)	2 (3.85)		
Fever and vomiting	1 (1.92)	1 (1.92)		

The article "Effects of Ulinastatin on Myocardial Ischemia-Reperfusion Injury, Cardiac Function, and Serum TNF-α and IL-10 Levels in Patients Undergoing Cardiac Valve Replacement under Cardiopulmonary Bypass" was retracted in 2023. Reasons: signs of a paper mill; suspected computer-generated content; unreliable results or conclusions; concerns about the data.

## Data Availability

The labeled dataset used to support the findings of this study are available from the corresponding author upon request.
